# A Clinical Study of the Effect of Estradiol Valerate on Sleep Disorders, Negative Emotions, and Quality of Life in Perimenopausal Women

**DOI:** 10.1155/2021/8037459

**Published:** 2021-10-16

**Authors:** Jianfu Zhang, Shurong Shao, Chaohui Ye, Bengui Jiang

**Affiliations:** ^1^Department of Pharmacy, Ningbo Women and Children's Hospital, Ningbo 315012, China; ^2^Department of Gynecology, Ningbo Women and Children's Hospital, Ningbo 315012, China

## Abstract

In this prospective study, we randomly divided 100 patients with perimenopausal syndrome equally into the control group (*n* = 50) receiving conventional treatment and the study group (*n* = 50) receiving estradiol valerate. The indicators observed were endometrial thickness, uterine volume, and the levels of LH (luteinizing hormone), FSH (follicle-stimulating hormone), and E2 (estradiol) of the patients before and after treatment. The Pittsburgh Sleep Quality Index (PSQI), Hamilton Anxiety/Depression Scale (HAMA/HAMD), Kupperman symptom score, and menopause-specific quality of life (MENQOL) were also applied to assess the sleep quality, negative emotions, severity of the condition, and quality of life of all patients, respectively. Our findings were that estradiol valerate is beneficial in improving serum sex hormone levels, sleep disturbances, negative mood, and quality of life in patients with perimenopausal syndrome and that its safety profile is high enough to warrant clinical promotion.

## 1. Introduction

With the advent of an aging society, a significant upward trend is being seen in the number of perimenopausal women. There are 850 million women aged 40–60 years globally, of which about 88% will experience perimenopause [1]. Perimenopausal syndrome is a group of symptoms associated with autonomic nervous system dysfunction and endocrine dysregulation, mostly caused by fluctuations and decreases in female sex hormones around the time of menopause, commonly in middle-aged women aged 45 to 55 years [2–4]. In a survey, 32.8% of perimenopausal women regained their balance through a neuroendocrine regulation mechanism, while the remaining perimenopausal women experienced perimenopause syndrome symptoms due to a decline in their sex hormone levels, which mainly manifested as psychological, endocrine, and metabolic changes [5, 6]. In addition, perimenopausal women often suffer from sleep disorders such as insomnia and abnormal rhythms, which can persist until late menopause and lead to concomitant symptoms such as vascular tension symptoms, anxiety, depression, and cognitive decline, which in turn have a serious negative impact on patients' quality of life [7–9]. Hormone therapy is one of the common ways of clinical treatment of menopausal syndrome [10]. Data show that hormone therapy can not only improve women's estrogen levels, reduce physical, and mental disorders but also help reduce the incidence of cardiovascular diseases [11]. Estradiol valerate is a long-acting estrogen preparation that can be used as a supplemental treatment for inadequate estrogen levels. This study mainly explored the effect of estradiol valerate on the improvement of sleep disorders in perimenopausal women and the impact on patients' bad mood and quality of life. A reference for the hormone supplementation therapy in patients with perimenopausal syndrome is provided, which is reported below.

## 2. Methods and Information

### 2.1. Clinical Data

One hundred patients with perimenopause syndrome diagnosed and treated in our hospital from June 2019 to June 2021 were selected for this study. Using a random number table, the patients were randomly divided into study and control groups, with 50 cases in each group. This study was approved by the medical ethics committee of our college (approval number EC2020-009).

### 2.2. Inclusion Criteria

Patients who met the relevant diagnosis in *Obstetrics and Gynecology*; patients aged 45 to 55 years; patients with a disease course of 2 to 4 years; patients with clinical symptoms such as hot flashes, sweating, insomnia, and anxiety, among which the menopausal time of the postmenopausal patients was less than 1 year; patients without contraindications to the drugs used in this study; and patients who signed an informed consent form.

### 2.3. Exclusion Criteria

Patients who were suffering from hypertension, diabetes, thrombotic diseases, gynecological malignancies, breast tumors, and other diseases, as well as endometriosis with obvious signs and symptoms; patients who were suffering from severe or unstable physical diseases or taking sex hormone preparations or health medications for the treatment of perimenopausal symptoms in the previous month; patients with severe mental illness or allergies; patients with severe infections or abnormal liver and kidney function; patients with anemia or primary hypotension; and patients with ovarian cysts or premature ovarian failure.

### 2.4. Treatment Programs

All patients receive health education, which require patients to maintain a good mental state and eating habits, cultivate interests that are conducive to physical and mental health, make their lives colorful, and participate in more personal physical exercises to promote blood circulation through exercises to improve symptoms of menopause. Patients in the control group were given oral oryzanol tablets (Anhui City Pharmaceutical Co., Ltd., Zhunzi H34020623) 1 tablet/time, 1 time/d, for 28 days of medication for 1 cycle, drug withdrawal for 7 days, and continuous treatment for 3 cycles. Patients in the study group were given oral estradiol valerate tablets (DEL PHARM Lille S.A.S H20160679) 2 tablets/d on the basis of patients in the control group, continuously taking 21 d, stopping the drug for 7 d, and 28 d as a course of treatment, continuously taking 3 courses.

### 2.5. Observation Index

Uterine volume and endometrial thickness: before and after treatment, the color Doppler ultrasound was used to detect the endometrial thickness and uterine volume of the two groups.

  Sex hormone levels: before and after treatment, 4 ml of fasting peripheral blood was drawn in the early morning in both groups, and the supernatant was collected after anticoagulation and centrifugation and placed in the refrigerator for inspection. The automatic chemiluminescence immunoassay instrument (model E170) and its kit (provided by Roche) were used to detect luteinizing hormone (LH), follicle-stimulating hormone (FSH), and estradiol (E2) level.
  Sleep quality: before and after treatment, the Pittsburgh Sleep Quality Index (PSQI) was used to evaluate sleep quality. The PSQI included 7 indicators of falling asleep time, sleeping time, sleep efficiency, sleep quality, sleep disorders, day dysfunction, and hypnotic drugs, each with a 0∼3 point scoring system, with a full score of 21 scores, and a total score of ≤7 was divided into normal sleep, and >7 points meant there was sleep disturbance.
  Negative emotions: before and after treatment, the Hamilton Anxiety Scale (HAMA) and Hamilton Depression Scale (HAMD) were used to compare the negative emotions of the two groups. A score system of 0∼4 scores was adopted. The total score of HAMA/HAMD > 20 indicated that the patient had mild to moderate anxiety/depressive symptoms, and the score >35 indicated that the patient had severe anxiety/depression.
  Kupperman symptom score: before and after treatment, the Kupperman symptom score was compared. It Included 12 items such as insomnia, fatigue, hot flashes and sweating, and irritability. A score system of 0∼3 scores was adopted, with a total score of 36 scores; the higher the score, the more severe the symptoms of menopausal syndrome.
  Quality of life: before and after treatment, the quality of life of the patients before and after treatment was evaluated using the menopause-specific quality of life (MENQOL). It included 4 domains of environment, psychology, physiology, and social relationship, and 2 overall evaluation items, totaling 26 items. Among them, positive entries were scored from 1∼5 and negative entries were reverse scored, with a total score of 0∼110; the higher the score, the higher the quality of life.
  Efficacy and safety: the clinical efficacy and various adverse reactions that occurred during treatment were compared between the two groups of patients. The treatment efficacy evaluation criteria are as shown in Table 1. Total effective cases = (recovery + remarkable effect + effective) cases.

### 2.6. Statistical Analysis

SPSS 24.0 statistical software was used to analyze and process the data, and GraphPad version 8 was used to draw the resulting graph. A chi-square test was used to count the data, and the measurement data were expressed as mean ± standard deviation. An independent-sample *t*-test was used for the intergroup comparisons, and a paired *t*-test was used for the intragroup comparisons. The rank sum test was used to grade the data. *P* < 0.05 was considered to be a statistically significant difference.

## 3. Results

### 3.1. Baseline Data Comparison

No significant difference was found between the two groups when comparing the patients' age, BMI (body mass index), smoking history, and drinking history and the course of perimenopause syndrome (*P* < 0.05, Table 2).

### 3.2. Endometrial Thickness and Uterine Volume

Before and after treatment, there was no statistical difference in endometrial thickness and uterine volume in the two groups (*P* < 0.05, Figure 1).

### 3.3. Hormone Levels

Before treatment, there was no significant difference in the levels of serum LH, FSH, and E2 between the two groups (*P* < 0.05). After treatment, the levels of LH and FSH in the two groups were significantly lower than those before treatment, and the levels of E2 were significantly higher than those before treatment, and the study group changed significantly compared with the control group (*P* < 0.05, Figure 2).

### 3.4. Sleep Quality

Before treatment, there was no statistical difference in PSQI scores between the two groups (*P* < 0.05). After treatment, the PSQI scores of the two groups decreased significantly, and the study group improved significantly compared with the control group (*P* < 0.05, Figure 3).

### 3.5. Negative Emotions

Before treatment, there was no significant difference in HAMA and HAMD scores between the two groups (*P* < 0.05). After treatment, the HAMA and HAMD scores of the two groups decreased significantly, and the study group improved significantly compared with the control group (*P* < 0.05, Figure 4).

### 3.6. Kupperman and MENQOL Scores

Before treatment, there was no significant difference in Kupperman symptom and MENQOL scores between the two groups (*P* < 0.05). After treatment, the Kupperman symptom and MENQOL scores of the two groups decreased significantly, and the study group improved significantly compared with the control group (*P* < 0.05, Figure 5).

### 3.7. Clinical Efficacy

The improvement in the clinical efficacy of the treatment was significantly higher among the patients in the study group than that among the patients in the control group (*P* < 0.05, Table 3).

### 3.8. Adverse Reactions

No significant difference was evident in the incidence of nausea, vomiting, breast pain, and a rash between the two groups (*P* < 0.05, Table 4).

## 4. Discussion

At present, the aging of the global population is becoming more and more serious. It is reported that women will spend one-third or more of their time in perimenopausal and menopausal periods [12]. The patient's clinical symptoms are mainly manifested in changes in psychology, endocrine, metabolism, etc., and this change can continue until the patient's menopause [13]. Specifically, the mental health of women with perimenopausal syndrome is generally poor, which has become a social problem, bringing a certain burden to the family and society. In addition, according to a 2005 study by the National Institutes of Health, about 39% to 47% of perimenopausal women have sleep disorders, and the proportion of menopausal women is as high as 60% [14]. Studies [15, 16] also show that prolonged sleep disturbance can cause many adverse reactions; for example, lack of sleep can lead to the accumulation of *β*-amyloid in the brain; long-term insomnia may reduce the prefrontal cortex and parietal gray matter of the brain capacity; and sleep disturbance can cause cognitive impairment or increase the incidence of Alzheimer's disease. It can be seen that sleep disorders not only affect the quality of life of perimenopausal and postmenopausal women but also endanger their lives and health in the long run and cause social burdens. This study found that estradiol valerate can effectively improve the clinical symptoms of perimenopausal diseases without increasing the adverse reactions of patients. It is expected to become a potential clinical treatment method.

In this study, we used estradiol valerate to treat patients. Estradiol valerate is an estrogen derivative, and its combined use with progesterone can supplement estrogen deficiency, maintain estrogen levels in the body, avoid the occurrence of neuropsychiatric symptoms, and relieve clinical symptoms such as sleep disorders and neurasthenia [17, 18]. In perimenopausal women, the level of hormones secreted by the ovaries changes significantly, causing uneven texture and reduced thickness of the endometrium [19]. In this study, we found that there was no difference in uterine volume and endometrial thickness between the two groups of patients after treatment. This shows that long-term use of estradiol valerate has little effect on women with perimenopausal symptoms and will not increase the incidence of endometrial cancer and breast cancer in women with perimenopausal symptoms.

It has long been clearly pointed out in clinical practice that ovarian function weakening can occur in perimenopausal women, which can cause a decrease in E2 and FSH and other estrogen. When hormone secretion is affected by degenerative diseases, it will cause neuroendocrine disorders and induce perimenopause syndrome [20, 21]. In this study, we also found that treatment with estradiol valerate significantly improved the levels of LH, FSH, and E2 hormones in the study group compared with the control group. The reduction of estrogen and its receptors in perimenopausal patients can also lead to dysfunction of the hypothalamic-pituitary-ovarian axis, and insomnia is one of the most common symptoms [22]. Sleep disorders not only affect the quality of life of women in the perimenopausal and postmenopausal periods but also endanger their lives and health in the long run, causing social burdens [23]. At the end of this study, we found that estradiol valerate improved the patient's sleep quality. In a study by Silva et al. [24], it was found that the sleep quality of patients treated with estradiol and trimesterone or after treatment was significantly higher than that of patients treated with placebo. This is similar to the results of our research. This also shows that estradiol can effectively improve the sleep quality of perimenopausal patients.

Besides, perimenopausal anxiety disorder is a disease in which women have anxiety manifestations during the perimenopausal period [25]. Perimenopausal women have autonomic nervous system disorders, and they will show negative mentality, irritability, restlessness, easy temper, insomnia, heart palpitations, long-term negative emotions, and easily aggravated depression and even display willingness to commit suicide; in severe cases, it is life threatening [26]. Kupperman symptom score and MENQOL score are clinically important scores for the condition and quality of life of perimenopausal patients [27, 28]. In this study, we found that the HAMA and HAMD scores of patients after treatment with estradiol valerate were significantly lower than those of the control group; the Kupperman symptom score and MENQOL score of the study group of patients were significantly higher than those of the control group. This shows that the use of estradiol valerate can improve the negative emotions and condition of perimenopausal patients and improve the quality of life of patients. Analyzing the reason, this may be related to the improvement of endocrine disorders in the patient's body after estradiol valerate treatment; insomnia, dizziness, hot flashes, lack of energy, irritability, and other symptoms are alleviated, so that the quality of life can be effectively improved [29].

In this study, we have determined through experiments that estradiol valerate can effectively improve sleep disorders in perimenopausal women, relieve bad emotions, and improve the quality of life. However, this study still has some limitations. First, there are fewer samples in this study. Secondly, we did not conduct long-term follow-up, and the long-term role of estradiol valerate in perimenopausal women is still unclear. We hope to verify our results through large-scale retrospective studies and long-term follow-up in subsequent studies.

In summary, estradiol valerate can improve sleep disorders in perimenopausal women, regulate the level of hormones in patients, relieve bad mood, and improve the quality of life of patients. It is worthy of clinical promotion.

## Figures and Tables

**Figure 1:** Uterine volume and endometrial thickness before and after treatment in the two groups. (a) Comparison of endometrial thickness between the study group and control group. (b) Comparison of uterine volume between the study group and control group.

**Figure 2:** Changes of hormone levels in two groups. (a) Comparison of LH levels between the study group and control group. (b). Comparison of FSH levels between the study group and control group. (c) Comparison of E2 levels between the study group and control group. Also, a was compared with the same group before treatment, *P* < 0.05<; b was compared with the control group after treatment, *P* < 0.05.

**Figure 3:** Comparison of PSQI scores between the two groups. a was compared with the same group before treatment, *P* < 0.05; b was compared with the control group after treatment, *P* < 0.05<.

**Figure 4:** Changes of HAMA and HAMD scores in the two groups. (a) Comparison of HAMA scores between the study group and control group. (b) Comparison of HAMD scores between the study group and control group. a was compared with the same group before treatment, *P* < 0.05; b was compared with the control group after treatment, *P* < 0.05.

**Figure 5:** Changes of the Kupperman symptom score and mental score in the two groups. (a) Comparison of Kupperman symptom scores between the study group and control group. (b) Comparison of mental scores between the study group and control group. a was compared with the same group before treatment, *P* < 0.05; b was compared with the control group after treatment, *P* < 0.05.

**Table 1:** Treatment efficacy evaluation criteria.

Level	Evaluation criteria
Recovery	The symptoms disappeared completely, hormones reached normal levels, and the Kupperman score decreased by more than 80% compared with that before the treatment
Remarkable effect	The MENQOL score was below 10, the symptoms were significantly relieved, the hormone indexes tended to be normal, and the Kupperman score decreased by 50%–80% compared with that before treatment
Effective	The MENQOL score was <20 and >10, the Kupperman score decreased by 30%–50% compared with that before the treatment, and hormone levels improved
Invalid	The MENQOL score was above 30, the MENQOL score decreased by more than 30%, and hormone levels did not improve

**Table 2:** Comparison of the patients' clinical data.

Factor	Control group (*n* = 50)	Study group (*n* = 50)	*P* value
Age			
≤50 years (*n* = 56)	25	31	0.227
>50 years (*n* = 44)	25	19	
Course of perimenopausal syndrome			
≤3 years (*n* = 53)	28	25	0.548
>3 years (*n* = 47)	22	25	
BMI (kg/m^2^)			
≤22	15	9	0.160
>22	35	41	
Smoking history			
Yes	8	5	0.372
No	42	45	
History of alcoholism			
Yes	5	3	0.461
No	45	47	

**Table 3:** Comparison of the clinical efficacy of the treatment.

Group	Recovery	Remarkable effect	Effective	Invalid
Study group (*n* = 50)	18	22	6	4
Control group (*n* = 50)	12	20	8	10
*Z*-value	−2.008			
*P* value	0.045			

**Table 4:** Comparison of the patients' adverse reactions to the treatment.

Group	Nausea and vomiting	Breast tenderness	Rash
Study group (*n* = 50)	3	2	3
Control group (*n* = 50)	2	1	1
*χ* ^2^ value	0.210	0.344	1.042
*P* value	0.646	0.558	0.307

## Data Availability

The data used during the current study are available from the corresponding author.
